The article "Analysis of the Influence of Comprehensive Nursing Intervention on Vital Signs and Negative Emotions of Patients with Gastrointestinal Polyps Treated by Digestive Endoscopy" was retracted in 2023. Reasons: signs of a paper mill; compromised peer review; unreliable results or conclusions.

# Analysis of the Influence of Comprehensive Nursing Intervention on Vital Signs and Negative Emotions of Patients with Gastrointestinal Polyps Treated by Digestive Endoscopy

**DOI:** 10.1155/2022/5931588

**Published:** 2022-06-24

**Authors:** Yaer Shi, Jianzhong Sang, Yimao Sang

**Affiliations:** Department of Gastroenterology, Yuyao People's Hospital, Yuyao 315400, Zhejiang Province, China

## Abstract

This research sets out to elucidate the influence of comprehensive nursing intervention (CNI) on vital signs (VSs) and negative emotions (NEs) of patients with gastrointestinal polyps treated by digestive endoscopy. To address this, from January 2020 to February 2021, 92 cases of gastrointestinal polyps treated by digestive endoscopy in the Yuyao People's Hospital of Zhejiang Province were partitioned into two different groups: the control group (CG; *n* = 46) intervened by routine nursing intervention, and the research group (RG; *n* = 46) treated by CNI based on routine care. The VSs, NEs, time of first postoperative exhaust and defecation, early food intake, length of stay (LOS), quality of life (QOL), nursing satisfaction, and the incidence of postoperative complications were compared between groups. When entering the operating room, elevated systolic/diastolic (SBP/DBP) was observed in CG compared with RG (*P* < 0.05) while there was no statistical difference in SBP/DBP in RG before intervention and when entering the operating room (*P* > 0.05). Statistically, less time of first exhaust and defecation as well as LOS and early food intake were observed in RG (*P* < 0.05). The HAMA and HAMD scores declined in both arms postintervention, and the decrease was more obvious in RG (*P* < 0.05). After intervention, the scores of various domains of GQOLI-74 elevated in both arms, and the increase was more obvious in RG (*P* < 0.05). RG also showed a lower total complication rate and a higher degree of nursing satisfaction than CG (*P* < 0.05). CNI for patients with gastrointestinal polyps treated by digestive endoscopy can obviously relieve their anxiety and depression, with stable VSs, short LOS, and low incidence of complications.

## 1. Introduction 

Gastrointestinal polyp is a relatively common gastrointestinal disease in the clinic, which has certain cancers. Clinical research has reported that gastrointestinal polyps are responsible for most colorectal carcinoma, so timely surgical treatment should be performed to prevent the disease from progressing [1]. Besides, it has been confirmed that if the gastrointestinal polyps are too large, patients will suffer from gastrointestinal bleeding and other symptoms to a great extent, which will seriously threaten the life safety of patients [2]. At this stage, digestive endoscopy is widely used for minimally invasive treatment of gastrointestinal polyps in clinical practice. However, patients are prone to anxiety, irritability, and other negative emotions (NEs) during the whole perioperative period due to their lack of understanding of the surgical methods and symptoms like pain, which leads to a decrease in the treatment effect. Therefore, it is particularly important to adopt scientific and reasonable nursing methods [3].

In this paper, comprehensive nursing intervention (CNI) is patient-centered, which is a care model starting from patients' multiangles and multidimensions, and taking different intervention measures in different stages and aspects, aiming at achieving the purpose of comprehensive nursing. At present, this nursing model has been carried out in various departments such as orthopedics & obstetrics and has shown favorable nursing effects [4–6]. However, there is currently a paucity of studies regarding its impacts on the vital signs (VSs), NEs, and quality of life (QOL) of patients with gastrointestinal polyps treated by digestive endoscopy. Accordingly, this study selects 92 cases of gastrointestinal polyps treated by digestive endoscopy in our hospital as the research participants, discusses the influence of CNI on their VSs, NEs, QOL, and other aspects, and compares it with the conventional nursing model.

The remaining manuscript is prepared to confer to the succeeding memo items which are given as follows.

Data and methods, which are used in this article, are presented in the subsequent section whereas Section 3 is reserved for the discussion of various results collected through various experiments. Finally, the conclusion section is provided which consists of the summary of the whole paper.

## 2. Methods and Data

### 2.1. General Information

Prospectively, 92 patients with gastrointestinal polyps who were treated by digestive endoscopy in the Yuyao People's Hospital of Zhejiang Province between January 2020 and February 2021 were partitioned into two different groups: research and control groups (RG & CG; *n* = 46). Inclusion criteria were as follows: (1) those aged 18–75; (2) those who received endoscopic treatment; (3) those who voluntarily signed the informed consent form; (4) those with complete clinical data; (5) those without contraindications to the treatment. Exclusion criteria were as follows: (1) those with malignant tumor(s); (2) those with mental illness and communication disorders; (3) those with cognitive dysfunction or unable to complete the questionnaire alone; (4) those who cannot cooperate and participate in other research projects. The Ethics Committee at the Yuyao People's Hospital of Zhejiang Province ratified the study protocol.

### 2.2. Methods

Gastrointestinal polyps in both groups were treated with digestive endoscopy, as shown in Figures 1 and 2. Postoperatively, CG was given routine nursing, such as inquiring about medical history, preoperative preparation, diet care, medication guidance, and postoperative nursing. RG was given CNI: (1) Preoperation care: after admission, patients were warmly received first, and the related information of the department was introduced in detail to reduce strangeness. At the same time, the occurrence mechanism and disease progression were explained to patients and their families as well as the operation methods and precautions. Furthermore, in order to build patients' self-confidence, patients were told about the successful operation cases and the importance of mutual cooperation. Preoperative contraindications were also explained to patients, including fasting and water deprivation for 6 hours, so as to fully drain the gastrointestinal tract and facilitate smooth operation. (2) Intraoperative care: the nursing staff assisted the patient to be in the left lateral decubitus position with bent knees and gently hold the patient's hands at the same time, so as to reduce his/her tension and fear and lower the occurrence of stress reaction. Then, the electrode plate was connected correctly to assist the doctor to place the endoscope to reach the surgical site. During this period, the patient's heartbeat, pulse, and other VSs were closely watched [7]. (3) Postoperative care: patients and their families were informed that the diet for 1–3 days after the operation should be mainly liquid food, and after the gastrointestinal function gradually returns to normal, it can be gradually transitioned to semiliquid food (rice porridge, millet porridge, and egg flower soup) until a normal diet. During the postoperative recovery period, the patients were advised to increase protein intake, not to eat spicy, cold, stimulating food, or smoke cigarettes, to prevent irritation of the gastrointestinal tract. In the early postoperative period, patients were asked to stay in bed as instructed by the doctor and avoid strenuous activities during the period. (4) Discharge guidance [8]: patients were informed to regularly test blood glucose and blood pressure and to seek medical treatment in case of any abnormality. They were also reminded not to get angry during the postoperative recovery period but to maintain a good mood. In addition, they were asked not to overeat and eat regularly. The reexamination time for patients with villous polyps was 3–6 months, and for those with hyperplastic polyps, the review time can be appropriately extended.

### 2.3. Endpoints

#### 2.3.1. Primary Endpoints

1. VSs of both arms of patients were monitored and compared before and after the intervention, including alterations in systolic/diastolic blood pressure (SBP/DBP).
2. Clinical indices such as the time of first exhaust and defecation time, early food intake, and length of stay (LOS) were counted.
3. Patients' anxiety and depression were assessed before and 7 days after intervention using the Hamilton Anxiety Scale (HAMA) [9] and Hamilton Depression Scale (HAMD) [10], respectively. The degree of anxiety and depression became more serious with the increase in scores.

#### 2.3.2. Secondary Endpoints

1. The Generic Quality of Life Inventory-74 (GQOLI-74) [11] was used for QOL assessment of patients before and 7 days after intervention from four aspects of social, physical, and psychological functioning as well as material life state. The scores of the first three dimensions range from 20 to 100 points, and the score of the last one is 16–80 points. The total score was proportional to the QOL.
2. The complications of the two groups were matched, including incision infection, bleeding, intestinal dysfunction, abdominal pain, and perforation.
3. In these groups, patients' nursing satisfaction was compared using the scale of self-made satisfaction of nursing [12] of the hospital. The scale included five parts: service attitude (10 points), diet and daily care (30 points), drug management (20 points), complications care (20 points), and clinical efficacy (20 points), with 100 points as the total score. Evaluation criteria were as follows: satisfaction (≥85 points), basic satisfaction (60–85 points), and dissatisfaction (<60 points).

(1) $$\begin{array}{c} \text{Satisfaction}=\frac{\left(\text{basic satisfaction}+\text{satisfaction}\right)\text{cases}}{\text{total cases}\times 100\%}. \end{array}$$

### 2.4. Statistical Processing

Data processing was performed by SPSS 20.0. Categorical data (*n*/%) were compared using the *χ*^2^ test. For quantitative data denoted by $\left(\bar{x}\pm s\right)$, intragroup (before and after treatment) and intergroup comparisons adopted paired *t-*test and independent *t*-test, respectively. Differences with *P* values <0.05 were considered to be of statistical significance.

## 3. Results

### 3.1. General Information

RG and CG were comparable in general baseline data such as gender, age, BMI, and disease type with no statistical significance (*P* > 0.05; Table 1).

### 3.2. Vital Signs (VSs)

The two arms showed no statistical difference in VSs related indexes before intervention (*P* > 0.05). When entering the operating room, elevated SBP and DBP were observed in patients in CG compared with RG (*P* < 0.05). In RG, SBP and DBP changed little before intervention and when entering the operating room (*P* > 0.05; Table 2).

### 3.3. Clinical Indices

The time of first exhaust and defecation, early food intake, and LOS were evidently shorter in RG than in CG (*P* < 0.05; Table 3).

### 3.4. Negative Emotions (NEs)

HAMA and HAMD scores showed no distinct difference between groups before intervention (*P* > 0.05). After the intervention, the two scores were reduced in both arms and were lower in RG versus CG (*P* < 0.05; Figure 3).

### 3.5. GQOLI-74 Score

RG and CG had no significant difference in the GQOLI-74 score before intervention (*P* > 0.05). After the intervention, the scores of various dimensions of the GQOLI-74 scale increased in both arms, especially in RG (*P* < 0.05; Table 4).

### 3.6. Complications

In RG, hemorrhage, intestinal dysfunction, and abdominal pain were observed in 1 case, 3 cases, and 1 case, respectively, with a total complication rate of 10.87% (5/46). In CG, there were 2 cases of incision infection, 2 cases of hemorrhage, 5 cases of intestinal dysfunction, 3 cases of abdominal pain, and 2 cases of perforation, with a total complication rate of 30.43% (14/46). An obviously lower incidence of complications was determined in RG compared with CG (*χ*^2^ = 5.370, *P*=0.021; Figures 4 and 5).

### 3.7. Nursing Satisfaction

With a satisfaction percentage of 93.48 percent, 20 cases in RG were satisfied, 23 instances were mostly satisfied, and three cases were unsatisfied. With a satisfaction percentage of 76.09 percent in CG, 15 instances were satisfied, 20 cases were mostly satisfied, and 11 cases were unsatisfied. In RG, nurse satisfaction was greater than in CG (*P*=0.020, 2 = 5.390; Figure 6).

## 4. Discussion

Gastrointestinal polyps are caused by multiple factors affecting the gastrointestinal mucosa of the body, which causes the epithelial part to bulge into the gastrointestinal cavity. Most patients complain of abdominal pain and discomfort as well as bloody stools [13–15]. At the present stage, endoscopic treatment is mostly used in clinical treatment. However, due to the lack of understanding of the surgical methods and preoperative notification of surgical risks, patients will eventually suffer from anxiety and other NEs, which lead to the reduction of cooperation degree and even serious stress reactions, resulting in unsmooth operation and poor treatment effects [16]. Some scholars have confirmed [17, 18] that taking scientific and reasonable nursing methods for patients undergoing surgery can obviously reduce the degree of anxiety, which can better contribute to the smooth operation, reduced complications, and accelerated postoperative rehabilitation of patients.

CNI is a nursing model based on advanced nursing concepts, starting from the patient and taking the patient as the center. This model carries out multifaceted development based on various intervention methods formulated in advance and provides sufficient psychological counseling for patients before surgery, so as to eliminate patients' irritability and fear to the greatest extent and encourage them to receive surgical treatment in the best state [19]. At present, CNI has been applied in many departments such as orthopedics & obstetrics, and neurosurgery because of its complete nursing elements and extensive coverage [20]. According to other researchers, when 138 patients with cervical polyps were given CNI, the therapeutic effect of the observation group was stronger, and the frequency of problems was much lower than the control group [21]. When patients entered the operating room, SBP and DBP were greater in CG than in RG; there was no discernible change in RG before intervention and when patients entered the operating room in this study. Besides, HAMA and HAMD scores were reduced in both arms after the intervention, especially in RG. It indicates that CNI for patients with gastrointestinal polyps treated by endoscopy can obviously relieve their anxiety and stress reactions. It may be that CNI allows professional psychologists or counselors to conduct psychological counseling on patients, which can greatly alleviate patients' anxiety, depression, and other unhealthy psychology. This is because CNI not only pays attention to patients' disease care but also emphasizes mental health: preoperative psychological counseling greatly alleviates patients' concerns about the risk of surgery and enables patients to master certain self-regulation methods, prompting them to actively mitigate their bad feelings, with the best mentality to face surgery [22]. The results showed that the time of first postoperative exhaust and defecation, early food intake, and LOS were shorter in RG than in CG. At the same time, the scores of various dimensions of the GQOLI-74 elevated in both arms after the intervention, especially in RG. Moreover, RG had a lower total complication rate and a higher nursing satisfaction. All these suggest that CNI for patients with gastrointestinal polyps undergoing endoscopic treatment can significantly improve the QOL of patients and is more conducive to recovery from the disease, which is similar to related research results [23, 24]. It may be that CNI is a targeted and holistic nursing mode centered on patients, which puts patients' health and comfort first. Meanwhile, it can enhance patients' tolerance during operation and ensure the high efficiency of operation by carrying out preoperative and intraoperative nursing. Postoperative care and discharge guidance are beneficial to the recovery of patients' gastrointestinal function, thus speeding up the recovery of body function and reducing the occurrence of complications, with high recognition among patients [25].

However, the sample size of this study is small, and the data were from a single center, so the influence of CNI on patients' long-term psychological state and QOL after operation still needs to be confirmed by later multicenter and larger sample research.

## 5. Conclusion

CNI is a nursing model based on advanced nursing concepts, starting from the patient and taking the patient as the center. To sum up, CNI for patients with gastrointestinal polyps treated by digestive endoscopy can obviously relieve their anxiety and depression and contribute to stable VSs, short LOS, and low incidence of complications, which is worth clinical application.

## Figures and Tables

**Figure 1:** Colon polyp.

**Figure 2:** Dissection of colonic adenoma.

**Figure 3:** Comparison of HAMA and HAMD scores between the two groups before and after the intervention. Note: *t*-test was used; ^∗^indicates *P* < 0.05 associated with that before intervention; # designates *P* < 0.05 associated with the control group.

**Figure 4:** Incidence of complications in the control group.

**Figure 5:** Incidence of complications in the research group.

**Figure 6:** Comparison of patient satisfaction between two groups. Chi-square test was used; # indicates *P* < 0.05 compared with the control group.

**Table 1:** General information matching of these groups (*n*, $\bar{x}\pm s$).

Indicators	Research group (*n* = 46)	Control group (*n* = 46)	*χ* ^2^/*t*	*P*
Gender (*n*)			0.040	0.824
Male	24	25
Female	22	21

Age (years old)	41.2 ± 3.2	40.9 ± 3.5	0.429	0.669
BMI (kg/m^2^)	21.15 ± 2.26	21.24 ± 2.23	0.192	0.848

Type of disease (*n*)			0.180	0.672
Intestinal polyp	18	20
Gastric polyp	28	26

*Note*. *χ*^2^: Chi-square test statistics; *t*: paired test statistics.

**Table 2:** Matching of the vital signs before & after the intervention $\left(\bar{x}\pm s\right)$ (mmHg).

Groups	Time	SBP	DBP
Research group (*n* = 46)	Before intervention	120.25 ± 8.24	79.88 ± 5.41
	When entering the operating room	121.33 ± 8.65#	79.91 ± 5.34#

Control group (*n* = 46)	Before intervention	121.38 ± 8.21	79.85 ± 5.36
	When entering the operating room	135.69 ± 7.04^*∗*^	89.23 ± 5.09^*∗*^

*Note*. *t*-test was used; ^*∗*^ indicates *P* < 0.05 compared with that before intervention; # indicates *P* < 0.05 compared with the control group.

**Table 3:** Assessment of the frequency of complications between these groups $\left(\bar{x}\pm s\right)$ d.

Groups	Time of the first postoperative exhaust	Time of the first postoperative defecation	Early food intake	Length of stay
Research group (*n* = 46)	2.3 ± 0.8	3.1 ± 0.9	2.5 ± 0.7	6.8 ± 0.4
Control group (*n* = 46)	3.7 ± 0.6	4.9 ± 0.5	4.0 ± 0.5	7.9 ± 0.9
*T*	9.496	11.858	11.826	7.575
*P*	<0.001	<0.001	<0.001	<0.001

*Note*. *t*-test was used; # indicates *P* < 0.05 compared with the control group.

**Table 4:** Comparison of GQOLI-74 scores between the two groups before and after intervention $\left(\bar{x}\pm s\right)$ points.

Groups	Time	Social functioning	Physical functioning	Psychological functioning	Material life state
Research group (*n* = 46)	Before intervention	72.63 ± 4.28	75.42 ± 5.21	70.43 ± 5.17	67.49 ± 5.31
	After intervention	83.59 ± 5.33^*∗*^#	85.56 ± 6.47^*∗*^#	78.99 ± 5.38^*∗*^#	77.18 ± 4.27^*∗*^#

Control group (*n* = 46)	Before intervention	73.62 ± 5.01	76.01 ± 6.02	71.12 ± 5.20	68.97 ± 5.30
	After intervention	79.74 ± 6.21^*∗*^	82.27 ± 5.98^*∗*^	75.37 ± 6.06^*∗*^	72.53 ± 4.19^*∗*^

*Note*. *t*-test was used; ^*∗*^ designates *P* < 0.05 matched with that before intervention; # specifies *P* < 0.05 likened with the control group.

## Data Availability

The labeled dataset used to support the findings of this study is available from the corresponding author upon request.
